RETRACTED

# Efficacy of Zn-Aspartate in comparison with ZnSO_4_ and L-Aspartate in amelioration of drought stress in maize by modulating antioxidant defence; osmolyte accumulation and photosynthetic attributes

**DOI:** 10.1371/journal.pone.0260662

**Published:** 2021-12-23

**Authors:** Qasim Ali, Muhammad Waqas Mazhar, Muhammad Ishtiaq, Abdullah Ijaz Hussain, Khizar Hayat Bhatti, Mehwish Maqbool, Tanveer Hussain, Humaira Khanum, Tauqeer Sardar, Mubashir Mazhar

**Affiliations:** 1 Department of Botany, Government College University Faisalabad, Faisalabad, Pakistan; 2 Department of Botany, Mirpur University of Science & Technology (MUST), Mirpur, Pakistan; 3 Director Central Hitech Lab, Government College University, Faisalabad, Pakistan; 4 Department of Botany, University of Gujrat, Gujrat City, Pakistan; Ghazi University, PAKISTAN

## Abstract

Human population is exceeding beyond the carrying capacity of earth resources and stresses like water shortage faced by the plants is jeopardizing the food security. Current research study was aimed to investigate the potentials of Zn-Aspartate (Zn-Asp), Zn-Sulphate (ZnSO_4_) and L-Aspartate (L-Asp) to be used as osmolytes and role of various levels of these chemicals in combating drought stress in maize plants in Punjab, Pakistan. Study was performed on two plots corresponding to drought and controlled environments. The lamina of maize plants was sprinkled row wise with various treatments including No spray (NS), water sprinkle (WS), sprinkle with ZnSO_4_ 0.25% and 0.50%, sprinkle with Zn-Asp 0.25% and 0.50% and Foliar sprinkle of L-Asp 0.5% and 1%, respectively. Role of major osmoprotectants and secondary metabolites was analyzed and positive changes were found in total soluble sugars (41.16), flavonoids (5387.74), tocopherol content (9089.18), ascorbic acid (645.27) and anthocyanin (14.84) conc. which assists in mitigating drought menace on maize. Shoot mineral ions (Ca, K, Zn, P, Mg and N) status of water stressed maize plants was also analyzed and it was found that application experimental dose enhanced their availability to crop. Physio-biochemical studies were performed on antioxidants enzymes like superoxide dismutase (SOD), peroxidase (POD), carotenoid content (CC), malondialdehyde, hydrogen peroxide, aspartate and free amino acid contents. The activity of SOD was increased by 28.5% and activity of POD was increased by 33.33% due to foliar applied 0.5% Zn-Asp under drought stress. Photosynthetic pigments (chlorophyll A, B and total chlorophyll content) analysis was also carried out in this study. It was found that conc. of different chlorophylls pigments increased (chl-A: 2.24, chl-B: 25.12, total chl: 24.30) which enhanced photosynthetic activity culminating into better growth and yield). The level of malondialdehyde and hydrogen peroxide decreased by 43.9% and 32.8% respectively on treatment with 0.5% Zn-Asp proving the efficacy of the treatment in drought amelioration. Study reveals that Zn-Asp induced modulations are far better than conventional sulphate salts in mitigating water scarce environment. Current study recommends the use of the Zn-Asp to meet the global food and agricultural challenges as compared to ZnSO_4_ and L-Asp due to its better drought amelioration properties. This research provides valuable informations which can used for future research and practical use in agriculture fields by indigenous and other people to enhance yield of maize to meet the food necessities of country.

RETRACTED

## Introduction

Food is one of the major and fundamental needs of human life on earth. Plants and primarily crop are which provide all of food and these are plants selected from wild on hit and trial basis and then cultivated for domestic as well as commercial needs. The rural areas of the developing countries rely on grain crops like wheat, maize, rice and millet and their food primarily almost 75% is obtained from these crops [1]. Pakistan has predominantly agriculture based economy and its 70% population is directly or indirectly linked with crops or its by-products. Wheat, maize and rice are major and prevalently cultivated crops in Pakistan for food/grain needs of local people. The purpose of research on which research hypothesis designed was to design such method which can address drought stress on maize crop. In this investigation “role of Zn-Aspartate in comparison with ZnSO_4_ and L-Aspartate on maize crop yield” was carried out using different parameters and recommend the best dose of Zn-Aspartate.

Maize crop is very prevalently used as food and other confectionary products making an integral role in human life. Maize contains different phytonyms starch (72%), protein (10%), and fats (4%). The 100 g of maize provides 365 Kcal. It is grown throughout the world with an amount of 717 million metric tons per year annually. The maize corns are used for source of starch, oil, glue, sweeteners, beverages, industrial and fuel ethanol types. The maize is third most crop in Pakistan and about 6.4% of the total grain demand in Pakistan is met by cultivation of maize and the maize has potential to yield grains twice higher than other grain crops. Maize is cultivated on more than 118 million hectares across the globe and the total production of maize is around 600 million metric tons. In Pakistan maize is cultivated on more than one million hectares with annual production of 3.5 million metric tons [2]. In Pakistan, people of rural and mountaineous areas primarily depend on maize and millet for food and fodder requirements. The yield of crop-maize in Pakistan has been increasing with rate of 5.38% per year since 1971 to 2020 and currently its yield was 7,800 thousand tonnes in 2020. However, per acre yield in rural and urban areas is decreasing gradually and may be affected more severely in coming years due to drought and other climate changes stress. The irrigation water in canal systems of Pakistan is also decreasing day by day. Similarly, about 17% of croplands across the planet are without appropriate irrigation facilities and face water shortage environment [2]. The decrease in river water, rainfall scarcity or pattern of raining has also been altered in Pakistan due to pollution and other climatic changes leading towards water scarcity and stress on plants and crops.

RETRACTED

Water scarce environment leads to reduction in ability of food factories of the plants to manufacture food as drought leads to closure of stomata and reduced activity of carbon fixation enzyme Rubisco [3]. The water drought is major culprit behind DNA fragmentation, reduction in stomatal conductance, lipid peroxidation and subsequently the cell death due to formation of Reactive Oxygen Species (ROS) which ultimately impart severe impact of growth and yield of the maize crop [4]. ROS leads to denaturation of enzymes and affect the functioning of plasma membrane by lipid peroxidation [5]. Water deficit environment leads to decrease in water potential and increase in the temperature of the leaf lamina thereby affecting photosynthetic attributes and reduction in yield [6]. The ROS may be in the form of super oxide radicals, peroxides and atomic oxygen. Generally, drought reduces the water potential of cropland and availability of the mineral elements from soil solution is retarded due to poor translocation however the foliar applied zinc is readily available to the plants for their efficient metabolism which is promulgation in various areas of world [7]. Similarly certain substances or antinutrients like phytate found in plant cells retard the normal process of absorption of minerals in the digestive tract of human being or livestock, which makes its less popular in food selection. Various techniques have been practiced worldwide for removal of phytates through fragmentation, modification, soaking and polishing however the removal of phytates has not been achieved completely. It is important to cultivate food crops and biofortify them with essential nutrients to achieve better results and prevention of antinutrients [8].

Plants have innate defense mechanisms to mitigate a short duration of drought and in response to production of ROS plants respond by producing various phytochemicals and osmolyte accumulation such as ascorbate and phenolics to combat environmental stresses [3]. The super oxide radicals induced by ROS are combated by antioxidant enzymes like superoxide dismutase (SOD) and activity of these enzymes is increased as internal plant defense mechanism becomes activated [9]. Controlling the formation of ROS by osmolytes in the form of treatment of plants with various enzymatic and non-enzymatic materials is a short term but effective strategy to control abiotic stresses [10]. Similar influence is noted by applying minerals and nutrients to the crops which enhance the plant metabolism [10]. The foliar sprinkle of various osmolytes and mineral nutrients is a prominent strategy for induction of drought tolerance and is comparatively better than soil amendments in form of fertilizers and other ingredients [11].

RETRACTED

Micronutrients play their part in cell wall formation, increasing plant immunity against pests and abiotic stressors. Zinc is an important nutrient and is activator of several enzymes like carbonic anhydrase, SOD, RNA and DNA polymerases, several types of dehydrogenases and aldolases are dependent on zinc for their functions [6]. Under drought and aridity conditions, topsoil absorbs less water and thus transport of zinc from soil solution to aerial parts of plants becomes difficult and challenging. Actually, Zinc deficiency means more accumulation of ROS in plants [9]. The antioxidant enzyme ‘SOD ‘requires copper and zinc for its proper functioning. The zinc availability is essential for integrity of biological membranes and is potential candidate in serving synthesis of biomolecules [12,13]. Over two billion people, among the current world population is vulnerable to zinc deficiency [14] and its deficiency is responsible for defects in male organogenesis process [13].

The living organisms contain nitrogenous compounds with organic nature called amino acids and these compounds polymerize to synthesize proteins. The same compounds act as starting materials for the synthesis of essential plant hormones like indole acetic acid (IAA) which is a growth booster [15]. Cereal like maize, wheat, rice and millets lack and are deficient on some occasions with certain specific amino acids. For instance, maize shows deficiency of lysine, tryptophan and methionine naturally and similarly wheat as well as rice lack lysine. These amino acids should be provided to the plants for regulation of metabolism and for better yield acquisition [16]. Amino acid ‘proline’ has been used as osmoprotectant to ameliorate drought stress losses [17]. Four amino acid which are essential for maize plants are derived from the biosynthetic pathways of aspartate. For human food, although the deficiency of amino acids is met by supplements obtained from animal food however the amino acids acquisition through cereal and millets is quite safe and productive [18].

RETRACTED

The combined effect of minerals and amino acids has long been thought to improve physiological and biochemical status of plants and for healthy membranes structure and functions [15]. The amino acids bear carboxyl group in their structure and minerals have close affinity for carboxyl ends of amino acids. Being very important building material and unique sort of nitrogenous compounds amino acids serve as better chelating agents in terms of performance; however there is still debate on how this chelation property of zinc with amino acids confers zinc adaptation for the regular functioning of plants [14].

Although zinc sulphate is an important traditional foliar spray that is applied to cereal to enhance their performance [7]. It has been found encouraging in improving photosynthetic capabilities of plants [19], however being saline in nature its application is still questionable in all types of soils. In the light of literature surfing and according to our knowledge very little is known about ‘effects of mineral chelated amino acids’ in increasing yield and inducing drought tolerance in plants. Although, zinc sulphate has been extensively supplied on various crops but keeping in view all circumstances, we hypothesize that “Zn chelated aspartate and aspartate acid might be more effective in reducing the adverse effects of water stress with increase in antioxidant defence, osmolyte accumulation and mineral acquisition patterns in comparison with ZnSO_4_”. The key objectives of the present study were to: (i) explore the ameliorating potentials of ZnSO_4,_ Zn-Asp and L-Asp sprays to mitigate drought menace,(ii) determine how much contents of chlorophyll are increased and how much conc. of different growth regulating enzymes conc. is increased or activated”. Water stress caused by drought is impeding parameter in growth as well as yield of maize crop in Pakistan and through this study we will recommend the best solution (recipes) for reclamation and improvement of maize crop production in the study area. This model experiment may also be employed for other parts of country and world for better yield production of maize crop.

## Materials and methodologies

### Experimental setup and design

Maize seeds with healthy form without any symptoms of diseases or stress were collected from agriculture research centre Faisalabad, Pakistan. The seeds were sown and maize plants were raised under open field conditions in form triplicate of experimental trials in Botanical Garden of Government College University Faisalabad. The study was divided into two major plots corresponding to control and stressed environment experimental trials involving split plot factorial design following protocol of Nasri, (2015) and Ram *et al*., (2016) [1,3]. Each of the plots was further classified into eight rows with respect to differential treatments. Twenty plants of maize were cultivated in each row. The soil was supplied with sufficient moisture at the time of seed plantation. Soil was silty clay loam having pH of 8.27, and EC 0.568. the amount of organic matter was 1.98%. To explore water moisture content or water holding capacity (WHC) of field analysis of soil was performed by taking three samples as in replica from of experimental soils. About 200g of soil samples was taken and weighed. Then it was dried in oven for 24 hours at 105°C temperature. After drying, soil samples were again weighed for quantification of soil moisture contents or WHC. The field capacity was calculated by applying following equation using protocol described by Khan *et al*., [12].

$$M.C.=(W_{nss\;‐}W_{ods})\;X\;100/W_{ods}$$

where, Wnss is weight of water in normal Soil sample measured in grams; Wods = weight of oven dried soil samples measured in grams; “nss” means normal soil sample and “ods” means oven dried soil.

RETRACTED

The research was designed and conducted in first week of August 2016. The seeds were obtained from Ayub Agriculture Research Institute, Faisalabad Punjab, Pakistan. Before plantation, the seed were subjected to surface sterilization with 0.1% mercuric chloride solution. Twenty seeds were sowed in each row as described above maintaining good soil moisture for root development. The germination of seeds was monitored carefully for raising a healthy crop. Periodic thinning and tillage was performed removing a total of five plants from each row and thus, distance between individual plants was found around 25 cm. The plants were given first proper irrigation during second week of germination. The subplot maintained under water stress was given water treatment on two occasions i.e. on vegetative and flowering stage. However, the plot under control label trial was given irrigation as per normal irrigation requirements. The plants were subjected to water shortage conditions from third week of germination. The experimental field trial plots were supplemented with animal manure at concentration of 125 Kg per hectare Ali *et al*., [19].

### Chelation synthesis and treatment application

The method given by Leu [20] was followed for the preparation of Zn and Aspartic acid chelate. Around 260 g ZnSO_4_.7H_2_O was weighed and dissolved in H_2_O, then L-aspartic acid monohydrochloride was weighed at 146.12 g and was added in water containing zinc salt. The mixture was heated at 95°C for 3 hours as per given protocol.

RETRACTED

The two concentrations (0.25% and 0.50%.) of each of Zn-Asp, ZnSO4 and L-Asp were prepared and applied on first row of experimental plot. The second row was given only water sprinkle keeping as control or standard. The leaf laminas of plants cultivated in third and fourth rows were sprinkled with 0.25% and 0.50% ZnSO_4,_ respectively_._ The fifth and sixth rows were treated with Zn-Asp solution having concentration of 0.25% and 0.50%, respectively. The seventh and eighth rows were given foliar spray of L-Asp with conc. of 0.25% and 0.50%, respectively. The treatment was employed on each of three (replica) experimental plot from 20 days of induction of drought stress. Then plants grown upto 110 days life were collected and stored at -80°C until used for further physio-biochemical analysis in laboratories.

### Analysis of photosynthetic pigments

Plant pigment (chlorophyll) contents have significant role in photosynthesis and growth as well as on yield of crop or any plant. Chlorophyll contents were analysed using the method of Arnon [21]. Freshly collected maize leaf (ca. 0.1g) were crushed in 5 mL of 80% acetone at 04°C. Then solution of acetone was filtered using Whatmann 42 paper and filtrate was used to determine chlorophyll contents. Ultraviolet visible spectrophotometry was performed by recording absorbance by each sample at 663 nm, 645 nm and 480 nm [21].

Amount of carotenoids was analysed using the formula described by Kirk and Allen [22]. Expression units used are mg/g fresh weight.

The chlorophylls ‘a’ and ‘b’ were calculated by the following formulae:

Chl.a=[12.7(OD663)–2.69(OD645)]×V/1000×W

Chl.b=[22.9(OD645)–4.68(OD663)]×V/1000×W

V = volume of the extract (mL)

W = weight of the fresh leaf tissue (g)

Total chlorophyll content were estimated by a total of chl. a and chl. b

Carotenoids (mg ml^-1^) = A.car/Em 100%* 100

A Car (carotenoid) = (OD 480) + 0.114 (OD663)-0.638(OD645)

Em (Emission) = Em 100% = 2500

### Extraction of antioxidant enzymes

Antioxidant enzymes were extracted from the leaf samples following different protocols for each enzyme which is described below. The leaf tissues (0.5g) were grounded by mortar and pestle in 5ml of 50mM chilling phosphate buffer. The mixture was filtered and centrifuged at 15000 rpm for 20 minutes at 4°C. Antioxidant enzymes’ conc. were studied using following procedures.

#### Superoxide Dismutase (SOD)

The SOD activity and conc. was determined using method of Giannopolitis and Ries [23]. One unit of SOD was considered equivalent to amount of enzyme that cause 50% inhibition in nitro blue tetrazolium (NBT) photoreduction when compared to blank (without enzyme extract). The reaction solution for SOD was prepared which contained 50 mM phosphate buffer (pH 7.8), distilled water, methionine 13 mM, NBT 50 μM, enzyme extract 50 μl and riboflavin1.3 μM. The reaction mixture was kept under 15 fluorescent lamps for 15 min and absorbance was measured at 560 nm using spectrophotometer.

RETRACTED

#### Peroxidase (POD) activities

Activity and conc. of POD was determined on protein basis by following the Chance and Maehly [24] method. For determination of POD activity, the reaction solution was prepared containing distilled H_2_O, 250 μl of 50 mM phosphate buffer (pH 7.8), 100 μl of 40 mM H_2_O_2_,100 μl of 20 mM guaicol and 50 μl enzyme extract. The change in enzyme activity was determined after every 20s at 470 nm through spectrophotometer apparatus.

### Analysis for oxidative stress indicators

#### Malondialdehyde (MDA) contents

MDA contents were noted by method described by Cakmak and Horst [25]. Fresh leaves of maize (1g) were homogenized in 3ml solution of 0.1% tricarboxylic acid (TCA). The mixture was centrifuged at 20000 x *g* for 15 min. Method involves the use of Thiobarbituric Acid (TBA). About 1 mL of grounded mixture was mixed with 4 mL of 20% TCA having 0.5% of TBA in a test tube. Test tubes containing these solns. were covered and kept in hot water bath at temperature of 95°Cfor40 minutes and then cooled immediately on ice for 5 minutes. The samples were again centrifuged at10, 000 ×*g* for 10 min. Absorbance was noted at 532 nm and 600 nm using a spectrophotometer. The MDA contents were calculated using extinction coefficient of 155/ (mm cm) 1) using the following formula:

MDA(nmol)=Δ(A532nm–A600nm)/1.56×105

#### Measurement of H_2_O_2_ contents

H_2_O_2_ contents were studied by using method given by Velikova *et al*., [26]. Test mixture was obtained by homogenizing0.1g of fresh leaf with 5 mL vol. 0.1% TCA on an ice bath. The extract was centrifuged at 12000 rpm for 5 minutes. Then about 0.5 mL of test extract and 0.5 mL of Potassium Phosphate Buffer was taken in a test tube in admixture form. Later on, 1 mL of 1 M Potassium Iodide solution was added in reaction mixture. Then finally mixture was shaken well before taking reading at 390 nm using a spectrophotometer.

### Determination of total soluble protein and free amino acids

#### Total soluble protein

Quantification of total soluble protein was performed by method given by Bradford [27]. About 0.5g of the plant tissue was grinded in 10 mL of phosphate buffer in chilling environment. The solution was centrifuged at 1000 rpm for 10 minutes. Later on, 1 mL of sample was mixed with Bovine Serum Albumin (BSA) also known as Bradford‘s reagent and absorbance from supernatant was measured at 595 nm using spectrophotometer.

RETRACTED

#### Free amino acid contents

Concentration of free amino acid was measured by using the method of Moore and Stein [28]. Mesophyll tissues (0.5 g) were extracted using 10 ml phosphate buffer in chilling environment 4°C. The extract was centrifuged at 12000 rpm for 15 minutes. About 1 mL each Pyridine (10%) and Ninhydrin (2%) was mixed with extract. Reaction mixture was taken in a test tube which were covered by a cotton plug and aluminium foil. The reaction mixture was kept in a hot water bath for 30 minutes and then absorbance was read 570 nm using a spectrophotometer.

### Determination of shoot minerals

Powdered samples were digested using sulphuric acid as described by Wolf [29]. Contents of different cations like Ca^+2^, K^+^, Mg^+2^ and zinc were determined by Atomic absorption spectrophotometer (Hitachi, Model 7 JO-8024, Tokyo, Japan). Phosphorus content was determined spectrophotometrically using Barton’s reagent. The content of (N) was determined using method as described by Bremner and Keeney [30] from the digested material.

### Analysis for vitamin status

#### Ascorbic Acid (AsA) contents (Vitamin C)

The contents of AsA were examined by using method given by Mukharjee and Choudhari [31]. In this analysis, about 0.25 g of maize leaves were grinded in 10 mL of 6% Trichloro Acetic Acid (TCA) solution. About 4 mL of leaf extract was mixed with 2 mL of 2% Dinitrophenyl Hydrazine solution. In this mixture, one drop of 10% alcoholic thiourea was added. Then mixture was heated for 20 min and cooled at room temperature. After cooling 5ml of 80% of H_2_SO_4_ (V/V) was mixed at 0°C. The absorbance ratio of mixture solution was read at 530 nm using a spectrophotometer. Concentration of AsA in extracted leaf sample was calculated from standard curve prepared using varying AsA standards.

#### Tocopherol analysis (Vitamin K)

Leaf tocopherol contents were quantified following the method of Hates *et al*., [32] with some modifications. Fresh leaf material (0.5 g) from each sample was homogenized in 10 mL of a mixture of petroleum ether and ethanol (2:1.6, v/v) and centrifuged at 10,000 x *g* for 20 min. To 1 mL of aliquot, 200 μL of 2% 2, 2-dipyridyl in ethanol were added, agitated well and kept in dark for 5 min. Then 4 mL of distilled and deionized H_2_O were added to mixture and mixed well. The reading was taken at 520 nm using spectrophotometer. The tocopherol content was calculated using a standard curve prepared with known concentrations of α-tocopherol.

RETRACTED

### Flavonoids determination

#### Analysis for Total Flavonoids Contents (TFC)

Total flavonoid concentration (TFC) in mesophyll samples was studied following method illustrated by Karadeniz *et al*., [33]. One gram (1 g) of freshly collected leaves from each treatment sample plants were homogenized with 20 mL of 80% aqueous methanol in a mortar and pestle. The solution was filtered using filter paper (Whatman No. 42) and o.5 mL of filtrate was mixed with 3 mL of distilled water and 0.3 mL of 5% NaNO_2_soltuion. The admixture was vortexed and allowed to stand at room temperature for 5 min. Later on, 0.6 mL of 10% AlCl_3_ was added in this mixture solution. After 6 min, 2 mL of 1 M NaOH was added to the test tube and its volume was raised up to 10 mL by adding dist. Water. The absorbance of different solutions was measured by taking its absorption reading at 510 nm through spectrophotometer. Flavonoid contents were then studied using a standard calibration curve, prepared from rutin by use of spectrophotometer.

#### Anthocyanin estimation

For estimation of anthocyanin contents protocol of Velikova *et al*., and Nakata *et al*., [26,32] were followed in which 250 μL of acidic methanol (1% HCl, w/v) was used for grinding 50 mg fresh leaves of maize. Mixture was treated with low temperature at 4°C with stirring. Mixture was centrifuged 14000 rpm at room temperature for 5 min. Absorbance was measured at 530 nm and 650 nm by Spectrophotometer. Following formula was used to estimates the anthocyanin contents.

QAnthocyanin=(A530‐0.25×A657)×M‐1,

where Q Anthocyanin is corrected absorption value linearly correlated with number of anthocyanins, A 530 nm and 657 nm is the absorption at the indicated wavelength and M is the weight of plant material used for extraction (g).

### Analysis of sugar osmolytes

#### Total soluble sugars

Total soluble sugar contents were measured using Anthrone reagent by following methodology of Shahri *et al*., [19,33]. The Anthrone reagent was freshly prepared by using 200 mg of anthrone in 100 mL of conc. H_2_SO_4._ A volume of 250 μ L of acidic methanol (1% HCl, w/v) was used for grinding the 0.1g fresh leaves of maize. Mixture was kept at 4°C and centrifuged (14000 rpm at room temperature for 5 min). About 0.2 mL of enzyme extract was taken in a test tube and distilled water was added to bring volume upto 1 mL forming a test solution. To 0.1 mL of test solution, 3 mL of anthrone reagent was added. Test tubes were covered and placed in hot water bath for 10 minutes at 90°C. Mixture was cooled at room temperature and absorbance was measured at 625 nm using a Spectrophotometer.

RETRACTED

#### Reducing and non-reducing sugars

Reducing sugar contents were analyzed by using Dinitro Salicyclic Acid (DNS) reagent, a method described by Wood and Bhat [34].

#### Preparation of DNS reagent

DNS reagent was prepared according to Coughlan and Moloney [35]. About 10 g of dinitrosalicylic acid (DNS) and 300 g of sodium potassium tartrate (Rochelle salt) was added to 800 mL of 0.5 N NaOH and was gently heated to dissolve the reagents. The volume was made up to 1.0 L with addition of distilled water. A volume of 250 μ L of acidic methanol (1% HCl, w/v) was used for grinding 50 mg fresh leaves of maize. Mixture was kept at 4°C and centrifuged (14000 rpm at room temperature for 5 min).About 1 mL of enzyme extract was taken in a test tube and 4 mL of DNS reagent was added to mixture. Then mixture was kept in water bath in boiling water bath for 5 min and then cooled at chilling temperature, subsequently. Absorbance was measured using spectrophotometer at 540 nm. Contents of non-reducing sugars were obtained by subtracting contents of reducing sugars from total soluble sugars.

Non-reducing sugars = Total soluble sugars-reducing sugars.

### Statistical analysis

The data obtained was subjected to descriptive statistics involving ANOVA application and has been tabulated and presented in the form of figures.

## Results

The maize crop has very important role in comprehending the food necessities of people of Pakistan. Particularly, people of rural areas totally depend on crops for their domestic life needs. Maize is grown in different parts of the country but it faces low yield problems and issues. The scarcity of water for irrigation is becoming worsen because rivers are becoming shallow and with low water reservoirs. The other solution of this plethora is to use fortification process to improve the yield and grain quantity as well as quality of cereal and other fruit plants. Different fortification sprays are known and here various combinations were tried and the best optimized fortification foliar sprays were recommended for better maize crop yield in drought stressed conditions.

### Impact of Zn-Asp on biosynthesis of photosynthetic pigments

Water shortage due to climate changes has led to poor coloration of maize leaves deciphering the anomalous development of plastids. The photosynthetic attributes were studied to comprehend the performance of applied foliar treatments and results have been presented in Fig 1 and Tables 1 and 3.

**Fig 1:** Effect of foliar sprinkled treatments of ZnSO4, Zn-Asp and L-Asp on status of photosynthetic pigments (A) Total Chlorophyll (B) Chlorophyll “A” (C) Chlorophyll “B” and (D) Carotenoid values of maize plants subjected to water stress in comparison with well-watered conditions (mean ± SE; n = 3).

RETRACTED

**Table 1:** Mean squares and *p* values from ANOVA of the data for Antioxidants and photosynthetic attributes and the nutrients in shoots of water stressed maize plants treated with foliar sprinkle of ZnSO_4_ and Zn-Asp and L-Asp (df @0.005).

Source	df	SOD		POD		Chl.A	
**Stress**	1	652.37***	0.00	652.37***	0.00	2.24***	0.00
**treatment**	7	1.129ns	0.36	1.129ns	0.36	2.36*	0.04
**WS X T**	7	1.23ns	0.31	1.238ns	0.31	2.351*	0.04
**Error**	32	0.007		7.76		0.034	
**Source**	df	**Chl. B**		**T.Chlo**		**CC**	
**Stress**	1	25.12***	0.00	24.30***	0.00	1.718ns	0.20
**treatment**	7	1.63ns	0.16	1.83**	0.04	0.98ns	0.46
**WS X T**	7	0.67ns	0.69	1.29ns	0.28	0.95ns	0.47
**Error**	32	0.24		0.30		1.59	

Key: ns: Non-significant, df degree of freedom, SOD Superoxide Dismutase, POD Peroxidase, Chl. A Chlorophyll A, Chl.B Chlorophyll B, T.Chlo Total Chlorophyll, CC Carotenoids Contents.

Total chlorophyll, chlorophyll ‘a’ and ‘b’ contents along with accessory pigments (carotenoid) values were significantly reduced upon exposure to water shortage scenarios (Table 3; Fig 1). The exogenous sprinkle with all treatments affected photosynthetic attributes of maize plants under study however increasing or decreasing effect has been noted to be treatment specific. Overall, 10% increase in Chlorophyll a, 22% increase in Chlorophyll b and 15.46% increase in carotenoids upon foliar treatment with 0.5% Zn-Asp was observed. The data suggests that overall performance of Zn-Asp has been found encouraging as compared to other treatments and Zn-Asp has been more ameliorative (2.78±0.25) as compared to other treatments in mitigating water shortage (Table 3).

### Exogenous applications of Zn-Asp solution

The Zn-Asp solution was prepared and used for exogenous use in form of foliar spray on leaf of maize plants. The data was tabulated and presented in graphical form as shown Fig 2 which described that behaviour and modulation of antioxidant enzymes in maize plants grown under water shortage and well irrigated conditions. Data presented in form Fig 2A depicts activity of Superoxide Dismutase (SOD), under drought and control conditions. The activity of SOD shows significant elevation upon exposure to drought stress (36±0.04). The SOD is one of major antioxidant enzymes which prevents the plants from different damages induced by Reactive Oxygen Species (ROS). Maximum increase in activity of SOD is shown by Zn-Asp treatments (36±0.04) proving its efficacy over all other treatments in combating drought stress. Maximum increase in antioxidant enzyme POD has been observed by applying Zn-Asp as compared with ZnSO4 and L-Asp (Table 2; Fig 2). The activity of SOD was increased by 28.5% and POD was increased by 33% upon foliar treatment with 0.5% Zn-Asp.

RETRACTED

**Fig 2:** Effect of foliar sprinkled treatments of ZnSO_4_, Zn-Asp and L-Asp on status of Antioxidant Enzymes (A) Superoxide Dismutase SOD (B) Peroxidase POD activities in maize plants subjected to water stress in comparison with well-watered conditions (mean ± SE; n = 3.

**Table 2:** Mean squares and *p* values from ANOVA of the data for physio-biochemical studies performed on water stressed maize plants treated with foliar sprinkle of ZnSO_4_ and Zn-Asp and L-Asp.

Variation Source	*df*	AsA	FAC	BAC	TSS	RS	NRS
**Water Stress (WS)**	1	645.27*** (.00)	14.84*** (.00)	2.82** (.0022)	41.16*** (.0000)	1.101ns (.3087)	6.23* (.0179)
**Treatment (T)**	7	4.02** (.0029)	4.15** (.0024)	0.64ns (.7190)	5.59*** (.0003)	4.62** (.0012)	6.42*** (.0000)
**WS X PT**	7	3.65** (.0052)	9.90*** (.0000)	2.83* (.0183)	3.99** (.0030)	3.36** (.0083)	1.154ns (.3558)
**Error**	32	0.01	0.001	0.85	0.025	0.06	0.09
**Variation Source**	***df***	**TSP**	**TC**	**FLA**	**H**_**2**_ **O**_**2**_	**MDA**	**FAA**
**Water Stress (WS)**	1	55.15*** (.0000)	9089.18*** (.0000)	5387.74*** (.0000)	11.41** (.0019)	2.40ns (.1312)	1.68** (.0033)
**Treatment (T)**	7	1.31ns (.2775)	25.73*** (.0000)	64.86*** (.0000)	2.28** (.0523)	8.49*** (.0000)	1.37*** (.0000)
**WS X PT**	7	8.90*** (.0000)	14.59*** (.0000)	7.34*** (.0000)	1.17ns (.3461)	9.59*** (.0000)	1.19ns (.2496)
**Error**	32	0.001	1.20	0.024	0.058	6.49	0.07
**Variation Source**	***df***	**Ca**	**K**	**Mg**	**N**	**P**	**Zn**
**Water Stress (WS)**	1	49103.33*** (.0000)	4466.49*** (.0000)	921.57*** (.0000)	3130.79*** (.0000)	1631.57*** (.0000)	1744.21*** (.0000)
**Treatment (T)**	7	110.58*** (.0000)	5.64*** (.0000)	129.69*** (.0000)	15.45*** (.0000)	28.67*** (.0000)	10.65*** (.0000)
**WS X PT**	7	3.71** (.0047)	2.52** (.0345)	4.77*** (.0009)	4.42** (.0016)	4.19** (.0022)	6.41*** (.0001)
**Error**	32	0.09	0.23	0.01	0.33	0.012	0.001e

ns: Non-significant, df degree of freedom, AsA Ascorbic Acid, Asp Aspartate, TAC Total Anthocyanin, FAC Free Anthocyanin, BAC Bound Anthocyanin, TSS Total Soluble Sugar, RS Reducing Sugars, NRS Non Reducing Sugars, TSP Total Soluble Protein, TC Tocopherol Contents, FLA Flavonoids, SOD Super Oxide Dismutase, POD PerOxide Dismutase, FAA Free Amino Acid, Ca Calcium, K Potassium, Mg Magnesium, N Nitrogen, P Phosphorus and Zn Zinc

*, ** and *** = significant at 0.05, 0.01 and 0.001 levels, respectively.

The POD family of enzymes is known to be relevant to hydrogen peroxide levels which assist by converting H_2_O_2_ into water and oxygen thereby improving water relations.

RETRACTED

### Effect of Zn-Asp solution in depressing level of oxidative stress

It was found that levels of Malandialdehyde (MDA) were increased sharply upon exposing the maize plants to water shortage environment (Fig 3). The MDA is a major product of lipid peroxidation due to abiotic stresses. Various Foliar treatments of Zn-Asp solution did affect MDA levels, however by increasing or decreasing its conc.; the effect on oxidative stress is depressed. The maximum effect in decreasing levels of MDA has been shown by Zn-Asp with 0.5%Zn-Asp treatment i.e., 43.9% and L-Asp and ZnSO_4_ treatments have been comparatively least effective, respectively. Data presented in Fig 3B describes impact of various treatments on level of hydrogen peroxide. The levels of hydrogen peroxide are higher in drought affected leaf samples as compared with samples without any stress. Exogenous treatment of the plants with Zn-Asp reduces the level of H_2_O_2_ and the best impact in lowering these levels has been shown by Zn-Asp by 0.25% (Tables 2 and 3) where 32.8% reduction in H_2_O_2_was determined in study.

**Fig 3:** Effect of foliar sprinkled treatments of ZnSO_4_, Zn-Asp and L-Asp on status of Oxidative stress indicators (A) Melondialdehyde MDA (B) Hydrogen peroxide contents of maize plants subjected to water stress in comparison with well watered conditions (mean ± SE; n = 3).

**Table 3:** Mean and standard error data of various variables followed in the current experiment under both drought and control environment.

**Treatment**	**Total Chl.**				**Chl. A**				**Chl.B**			
	**Drought**		**Control**		**Drought**		**Control**		**Drought**		**Control**	
	Mean	S.E	Mean	S.E	Mean	S.E	Mean	S.E	Mean	S.E	Mean	S.E
**NS**	2.61	0.09	3.08	0.19	1.71	0.01	1.91	0.02	0.89	0.11	1.17	0.21
**WS**	2.63	0.53	3.09	0.26	1.70	0.35	1.93	0.03	0.93	0.18	1.16	0.29
**0.25% ZnSO4**	2.65	0.25	3.19	0.12	1.76	0.07	1.92	0.01	0.89	0.20	1.27	0.14
**0.5% ZnSO4**	2.74	0.20	3.27	0.26	1.81	0.09	1.97	0.02	0.93	0.12	1.30	0.28
**0.25% -Zn-Asp**	2.82	0.07	3.57	0.37	1.86	0.01	2.16	0.04	1.00	0.08	1.41	0.42
**0.5% Zn-Asp**	2.87	0.34	3.6	0.45	1.88	0.03	2.18	0.02	1.09	0.36	1.42	0.48
**0.5% Asp-Acid**	2.78	0.25	3.42	0.18	1.82	0.07	2.06	0.02	0.96	0.18	1.36	0.20
**1% Asp-Acid**	2.81	0.63	3.48	0.22	1.84	0.17	2.10	0.03	0.97	0.48	1.38	0.25
**Treatment**	**SOD**				**POD**				**MDA**			
	**Drought**		**Control**		**Drought**		**Control**		**Drought**		**Control**	
	Mean	S.E	Mean	S.E	Mean	S.E	Mean	S.E	Mean	S.E	Mean	S.E
**NS**	28.00	0.15	17.97	0.00	39.00	0.01	17.97	0.00	21.20	0.19	13.52	0.46
**WS**	27.00	0.01	17.50	0.00	40.00	0.00	18.00	0.00	15.64	1.10	12.91	0.19
**0.25% ZnSO4**	28.10	0.03	17.12	0.00	44.00	0.00	17.12	0.00	12.12	0.85	11.02	1.50
**0.5% ZnSO4**	29.50	0.04	16.45	0.00	44.28	0.00	16.45	0.00	13.90	2.39	10.26	2.43
**0.25% -Zn-Asp**	32.00	0.05	22.00	0.00	48.00	0.00	29.00	0.00	10.24	0.83	9.64	1.83
**0.5% Zn-Asp**	36.00	0.04	23.00	0.00	52.00	0.00	27.00	0.00	11.89	1.48	8.41	0.81
**0.5% Asp-Acid**	31.00	0.00	17.00	0.07	43.00	0.00	23.00	0.00	12.94	1.93	7.03	0.03
**1% Asp-Acid**	31.00	0.03	18.00	0.00	44.00	0.00	25.00	0.00	11.23	1.06	10.48	2.51
**Treatment**	**TSP**				**FAA**				**Ca**			
	**Drought**		**Control**		**Drought**		**Control**		**Drought**		**Control**	
	Mean	S.E	Mean	S.E	Mean	S.E	Mean	S.E	Mean	S.E	Mean	S.E
**NS**	985.00	0.44	1191.00	0.00	3.34	0.02	1.09	0.00	6.80	0.00	11.4	0.11
**WS**	987.00	0.23	1172.50	0.00	3.26	0.02	1.13	0.03	6.95	0.02	11.77	0.01
**0.25% ZnSO4**	1043.00	0.32	1172.50	0.00	2.99	0.01	1.13	0.00	7.25	0.02	12.05	0.02
**0.5% ZnSO4**	1084.00	0.05	1192.50	0.01	2.93	0.00	1.22	0.00	7.32	0.05	12.10	0.05
**0.25% -Zn-Asp**	1113.00	0.09	1318.50	0.07	2.00	0.04	0.90	0.00	9.30	0.05	12.20	0.05
**0.5% Zn-Asp**	1137.00	0.08	1292.50	0.06	2.20	0.02	1.00	0.00	8.90	0.08	12.50	0.05
**0.5% Asp-Acid**	1090	0.08	1200.00	0.00	2.32	0.00	1.13	0.02	7.93	0.03	11.60	0.05
**1% Asp-Acid**	1100.00	0.00	1250.00	0.01	2.40	0.06	1.22	0.00	7.95	0.02	11.89	0.05
**Treatment**	Mg				N				P			
	Drought		Control		Drought		Control		Drought		Control	
	Mean	S.E	Mean	S.E	Mean	S.E	Mean	S.E	Mean	S.E	Mean	S.E
**NS**	2.60	0.05	3.25	0.08	34.25	0.14	40.00	0.57	4.32	0.07	5.45	0.02
**WS**	2.75	0.02	3.50	0.05	34.25	0.43	42.00	0.57	4.52	0.01	5.70	0.11
**0.25% ZnSO4**	2.85	0.02	3.65	0.08	35.75	0.14	45.50	0.28	4.67	0.01	5.85	0.02
**0.5% ZnSO4**	3.05	0.02	4.10	0.05	36.75	0.14	46.50	0.28	4.67	0.04	5.95	0.02
**0.25% -Zn-Asp**	3.32	3.13	4.77	0.08	39.91	0.05	49.70	0.11	5.00	0.02	7.00	0.04
**0.5% Zn-Asp**	3.67	0.01	4.86	0.14	41.75	0.14	51.85	0.02	4.65	0.14	7.25	0.02
**0.5% Asp-Acid**	3.27	0.01	4.70	0.05	37.00	0.57	45.35	0.08	4.70	0.11	6.30	0.05
**1% Asp-Acid**	3.17	0.01	4.78	0.02	36.00	0.57	45.75	0.02	4.95	0.02	6.50	0.05
**Treatment**	**Tocopherol**				**AsA**				**FAC**			
	**Drought**		**Control**		**Drought**		**Control**		**Drought**		**Control**	
	Mean	S.E	Mean	S.E	Mean	S.E	Mean	S.E	Mean	S.E	Mean	S.E
**NS**	60.50	0.28	45.00	0.57	254.00	0.19	180.00	0.07	1.66	0.05	1.43	0.02
**WS**	62.50	0.28	45.00	1.72	256.00	0.02	191.00	0.06	1.72	0.02	1.46	0.01
**0.25% ZnSO4**	66.00	0.57	42.00	0.57	262.00	0.02	194.00	0.07	1.76	0.03	1.49	0.00
**0.5% ZnSO4**	65.50	0.28	45.50	0.28	261.00	0.00	200.00	0.02	1.82	0.00	1.50	0.01
**0.25% -Zn-Asp**	69.50	0.28	53.00	0.57	276.00	0.16	204.00	0.02	1.95	0.02	1.58	0.01
**0.5% Zn-Asp**	68.50	0.28	51.00	0.57	275.00	0.01	205.00	0.02	1.96	0.02	1.55	0.01
**0.5% Asp-Acid**	67.00	0.57	42.50	0.86	263.00	0.04	190.00	0.02	1.87	0.01	1.53	0.02
**1% Asp-Acid**	65.50	0.28	48.50	0.28	262.00	0.04	195.00	0.03	1.87	0.00	1.56	0.00
**Treatment**	**Flavonoids**				**TSS**				**RS**			
	**Drought**		**Control**		**Drought**		**Control**		**Drought**		**Control**	
	Mean	S.E	Mean	S.E	Mean	S.E	Mean	S.E	Mean	S.E	Mean	S.E
**NS**	7.55	0.22	4.50	0.05	2.17	0.04	1.36	0.02	0.44	0.06	0.18	0.57
**WS**	7.85	0.02	4.51	0.10	2.23	0.08	1.47	0.00	0.49	0.03	0.23	0.00
**0.25% ZnSO4**	7.90	0.15	4.64	0.02	2.36	0.08	1.95	0.03	0.58	0.03	0.25	0.01
**0.5% ZnSO4**	7.93	0.03	4.71	0.11	2.47	0.10	1.83	0.00	0.66	0.00	0.24	0.00
**0.25% -Zn-Asp**	8.61	0.10	5.40	0.00	2.73	0.00	2.00	0.14	0.75	0.00	0.28	0.04
**0.5% Zn-Asp**	8.85	0.03	5.49	0.08	2.78	0.00	2.07	0.21	0.78	0.00	0.32	0.02
**0.5% Asp-Acid**	8.92	0.04	5.69	0.06	2.71	0.10	1.79	0.01	0.75	0.00	0.24	0.00
**1% Asp-Acid**	8.79	0.00	5.72	0.02	2.61	0.15	1.88	0.03	0.69	0.01	0.26	0.02
**Treatment**	**Carotenoids**				**H2O2**				**K**			
	**Drought**		**Control**		**Drought**		**Control**		**Drought**		**Control**	
	Mean	S.E	Mean	S.E	Mean	S.E	Mean	S.E	Mean	S.E	Mean	S.E
**NS**	0.09	0.00	0.06	0.00	3.52	0.03	1.38	0.04	22.00	0.28	34.70	0.11
**WS**	0.09	0.00	0.06	0.00	3.48	0.01	1.35	0.24	23.00	0.57	34.70	0.05
**0.25% ZnSO4**	0.10	0.00	0.06	0.00	3.20	0.01	1.39	0.08	26.00	0.57	37.00	0.02
**0.5% ZnSO4**	0.10	0.00	0.07	0.02	3.16	0.01	1.32	0.22	26.00	0.57	38.00	0.02
**0.25% -Zn-Asp**	0.11	0.00	0.07	0.00	2.43	0.02	1.18	0.01	28	0.28	40	0.014
**0.5% Zn-Asp**	0.11	0.00	0.07	0.00	2.35	0.02	1.10	0.37	29.00	0.14	41.00	0.05
**0.5% Asp-Acid**	0.10	0.00	0.07	0.00	3.08	0.02	1.28	0.00	27.50	0.21	38.00	0.02
**1% Asp-Acid**	0.10	0.00	0.07	0.00	3.01	0.03	1.36	0.01	28.00	0.00	39.00	0.14
**Treatment**	**Zn**				**BAC**				**NRS**			
	**Drought**		**Control**		**Drought**		**Control**		**Drought**		**Control**	
	Mean	S.E	Mean	S.E	Mean	S.E	Mean	S.E	Mean	S.E	Mean	S.E
**NS**	0.82	0.01	1.35	0.02	3.88	1.17	2.83	0.17	1.73	0.02	1.18	0.60
**WS**	0.81	0.02	1.40	0.01	3.95	0.22	2.88	0.96	1.74	0.11	1.24	0.00
**0.25% ZnSO4**	1.15	0.00	1.93	0.00	4.15	0.62	2.97	0.11	1.78	0.04	1.34	0.05
**0.5% ZnSO4**	1.25	0.00	2.05	0.04	4.29	0.16	2.96	0.24	1.81	0.10	1.59	0.00
**0.25% -Zn-Asp**	1.25	0.01	2.15	0.02	4.35	0.75	3.21	0.10	1.98	0.00	1.72	0.10
**0.5% Zn-Asp**	1.35	0.00	2.25	0.01	4.45	0.17	3.36	0.09	2.00	0.00	1.75	0.18
**0.5% Asp-Acid**	0.95	0.02	1.41	0.01	4.16	0.04	2.90	0.77	1.96	0.11	1.55	0.00
**1% Asp-Acid**	0.97	0.028	1.42	0.02	4.29	0.65	2.95	0.05	1.92	0.16	1.62	0.00

RETRACTED

### Impact of Zn-Asp spray on protein-amino acid ratio

The foliar spray of Zn-Asp solution is proving to be very useful and the data is presented in Fig 4B which showed that there is significant increase in free amino acid pool of maize plants subjected to water shortage environment as compared to control. There is significant reduction in total soluble protein (Table 3; Fig 4A) due to stress induced ROS accumulation and subsequent breakdown of proteins contributing to the free amino acid contents. Exogenous application of various treatments affect concentration of amino acids and protein accumulation, however the increasing or decreasing effect is treatment specific and every treatment produces specific effect. The Fig 4A and 4B suggest that the foliar application of Zn-Asp has been most beneficial in decreasing the free amino acid pool and these amino acids may become the part of proteins as suggested by the increase in soluble contents upon treating with Zn-Asp.

**Fig 4:** Effect of foliar sprinkled treatments of ZnSO_4_, Zn-Asp and L-Asp on status of (A) Total Soluble Proteins and (B) Free Amino Acids of maize plants subjected to water stress in comparison with well-watered conditions (mean ± SE; n = 3).

### Zn-Asp solution spray enhances shoot mineral acquisition

The mineral nutrition is of prime importance to the plants for proper growth and seed production. Present study includes the findings related to mineral nutrient acquisition patterns of maize plants raised under the influence of drought stress and treated under various regimes of Zn-Asp, ZnSO_4_ and L-Asp (Table 3; Fig 5). The maize plants upon exposure to drought stress were found to show mineral deficiency signs such as retarded growth, leaf narrowing, crinkling and discoloration.

**Fig 5:** Effect of foliar sprinkled treatments of ZnSO_4_, Zn-Asp and L-Asp on status of shoot minerals (A) Calcium (B) Potassium (C) Magnesium (D) Nitrogen (E) Phosphorus and (F) Zinc of maize plants subjected to water stress in comparison with well watered conditions (mean ± SE; n = 3).

This phenotypic effect has been interpreted by the data presented in the Fig 2. The contents of Nitrogen, Phosphorus and Potassium (commonly known as NPK) were decreased upon induction of drought stress (Table 3; Fig 5) similar result were observed for calcium, magnesium and zinc (Fig 5), respectively. Foliar applied 0.5% Zn-Asp causes maximum increase in Mg contents i.e24% whereas contents of Phosphorus increased by 8% and Nitrogen contents were increased by 4% upon foliar applied 0.5% Zn-Asp. The comparative study of various treatments reveals that mineral amino acid chelates are better in enhancing nutrient acquisition patterns and Zn-Asp treatments can prove to be potential candidates in improving mineral acquisition patterns as compared to other treatments.

RETRACTED

### Zn-Asp solution sprinkling increases vitamin Conc

The studies were performed to comprehend the level of vitamins tocopherol and ascorbic acid under water shortage environment. In maize crop. Plants accumulate certain metabolism boosters to cope with oxidative stress. The tocopherol contents and ascorbic acid value found elevated upon imposition of drought stress as shown in Table 3; Fig 6. Treatments given further enhance levels of these essential stress mitigators and metabolism boosters. Maximum increase has been found with Zn-Asp treatments (68.8±0.28) under both stress and controlled environments (Tables 2 and 3). Foliar applied Zn-Asp 0.5% increased the contents of tocopherol by 13% where as the contents of ascorbic acid were increased by 8.6%.

**Fig 6:** Effect of foliar sprinkled treatments of ZnSO_4_, Zn-Asp and L-Asp on status of Vitamin E and C (A) Tocopherol contents as Vitamin E (B) Ascorbic Acid Contents as Vitamin C of maize plants subjected to water stress in comparison with well-watered conditions (mean ± SE; n = 3).

### Zn-Asp solution increase Conc. of flavonoids and sugar osmolytes

Anthocyanin amount in the study trails proved that different levels of anthocyanin were being interpreted by Fig 7 and Tables 2 and 3; where data for free anthocyanin values and bound anthocyanin values has been given respectively. The figures show that induction of drought stress results in increasing the anthocyanin levels in maize plants. Increase in levels is part of innate defense behaviour under drought stress. The foliar applications of treatments (1.99±0.02) significantly enhance the levels of anthocyanin. Maximum increase in the anthocyanin values has been shown by Zn-Asp with increase of flavonoids by 17% and thus supporting the maize plants to withstand drought stress. Maize plants raised under drought conditions also cause significant increase in flavonoids. Zn-Asp treatment increases 17% increase in the levels of flavonoids and thus increased production of secondary metabolites favours the maize plants to overcome water shortage environment (Table 3; Fig 7).

**Fig 7:** Effect of foliar sprinkled treatments of ZnSO_4_, Zn-Asp and L-Asp on status of (A) Free Anthocyanin (B) Bound Anthocyanin (C) Total Flavonoids (D) Total soluble sugars (E) Reducing and (F) Non Reducing sugars of maize plants subjected to water stress in comparison with well-watered conditions (mean ± SE; n = 3).

Data presented in Fig 7D–7F is for the total soluble sugar levels, contents of reducing sugars and contents of non-reducing sugars respectively in maize plants raised under drought and controlled environment. Foliar sprinkling with various treatment affect the sugar levels of maize plants however the increasing or decreasing effect is treatment specific. Zn-Asp treatment causes maximum increase in the accumulation of these osmolytes enabling the maize plants to withstand drought stress (Tables 2 and 3). The levels of total soluble sugar increased by 28.6% upon foliar treatment with 0.5% Zn-Asp. Under all cases the Zn-Asp treatment is highly significant in increasing the contents and is better than ZnSO_4_.

RETRACTED

## Discussion

Current study highlights the significance of mineral amino acid chelates and proves the efficacy of Zn-Asp treatments over all other treatments to ameliorate ROS induced damages in plants upon induction of drought. The study was conducted to access various physiological and biochemical attributes of maize plants under the water shortage environment upon application of Zn-Asp and Zinc salts. Studies reported in past provide evidence about effectiveness of zinc salts in the forms of zinc sulphate in improving plant behaviour under the influence of the drought [17]. The mineral amino acid combination has been successful in a comparative study conducted on Ajwain by Ali *et al*., [36] proving the worth of mineral amino acid combination over all other treatments in the form of iron salts under the influence of the drought stress.

### Decrease in Solar Light Absorption (give key findings)

A fully developed chloroplast organelle has around 3000 constituent proteins. The structure and function of these proteins is affected negatively on drought induction and thus photosynthetic capabilities of the plants are affected [37]. The current study presents analysis of variance results to support that Zn-Asp treatment is best among all other treatments studied and analyzed here in raising the concentration of photosynthetic pigments and improving the photosynthetic potential of maize plants under the drought stress. The drought stress leads to poor carbon fixation due to stomatal closure and decreased activity of Rubisco [3]. About, 10% increase in Chl a, 22% increase in Chl b and 15.46% increase in carotenoids upon foliar treatment with 0.5% Zn-Asp was observed under drought stress. Plants accumulate pigments such as carotenoids under the increased influence of ROS as internal defense mechanism. The treatments of Zn-Asp causes further increase in the photosynthetic pigments and enhanced concentrations of total chlorophyll contents, chlorophyll a, chlorophyll b, and carotenoids. These results are in accordance with the recent work reported by Ali *et al*., [36] on Ajwain plants.

### Role of Zn enzyme

Activities of antioxidant enzymes speed up on arrival of stress conditions in plants as internal defense mechanism becomes active to cope with ROS formed as result of stress. In current study the SOD and POD activities were monitored under the influence of drought stress and found high. These results are supported by studies on antioxidant enzymes performed by Anjum *et al*., [17]. A further increase in the activity of SOD and POD was seen by foliar sprinkle with Zn-Asp indicating that plants show better defense mechanism under the influence of Zn-Asp with 0.5% Zn-Asp. The POD activities were also found to be increased under the influence of the drought stress. The POD family enzymes mitigate higher values of H_2_O_2_ raised under drought stress by converting it to water and oxygen [38]. The better activity of SOD and POD might be due to ample availability of Zinc supplied as treatment in the current study as zinc is activator for these enzymes.

RETRACTED

### ROS induced H_2_O_2_ formation and membrane lipids degradation

The drought causes lipids peroxidation and resultantly MDA accumulation is observed. More MDA means increased breakdown of membrane lipids. Maximum reduction in MDA concentration i.e. 43.9% was noted by Zn-Asp treatment. This reduction correlated the role of aspartic acid as a signalling molecule with lipid peroxidation [39]. The increased stress accumulates increased ROS and ROS induces the formation of H_2_O_2_. Foliar applied Zn-Asp lowers the ROS mediated formation of hydrogen peroxide by 32.8%.

### Supplying aspartate family amino acids by Zn-Asp application

A correlation of increase in free amino acid due to drought mediated proteins breakdown was also examined. Drought stress leads to degradation of proteins due to decreased concentration of growth hormones such as IAA. Zinc acts as important material in synthesis of IAA [15] and thus leads to increase in protein contents and subsequently decreased amino acid pool. Such results are the part of current study. Joshi *et al*., [16] reported that maize plants lack methionine, lysine and tryptophan amino acid. Four major and essential amino acids lysine, methionine, threonine and isoleucine find their biosynthetic pathway starting from aspartate [18]. In current study both zinc and aspartate were synergistically applied to meet the deficiency of these amino acids and better results were achieved by the Zn-Asp as compared to other treatments. The combination helps the plant to behave physiologically well under the drought stress.

### Improvement in cellular water levels by mineral uptake

The intensive cropping to meet the requirements of ever exceeding population of human has put the soil and croplands under the nutrient stress. Current study highlights that the contents of essential micronutrients (K, N, P, Mg, Ca and Zn) increase significantly upon treatment with Zn-Asp under the water shortage scenarios. These results are in accordance with a study performed on black gram by applying zinc [40]. The increase in minerals in maize plants under the influence of drought may be due to improved nutrient acquisition patterns due to application of metal chelated amino acid [41]. The amino acid metabolism improves cellular water relations as shown by *Codiaeum variegatum* L. plants when subjected to various levels of glutamic acid [38]. Current study highlights the significance of Zn-Asp as compared to all other treatments in improving mineral ion status of maize plants subjected to water shortage environment.

RETRACTED

### Vitamins provide stress mitigating support

Among vitamins, the vitamin C (ascorbic acid) and vitamin E (tocopherol) analysis was the part of current study. The contents of these components also show increased concentration upon induction of drought environment as a part of plant internal defense mechanism. The foliar application of Zn-Asp further raises the concentration of vitamin C (275±0.01) and vitamin E (68.5±0.28); thus supporting the plant internal defense against abiotic stressors.

### Accumulation of flavonoids and osmolytes for stress mitigation

The concentration of flavonoids is also enhanced under the influence of drought. Foliar sprinkle with Zn-Asp significantly increased the contents of flavonoids enabling the maize plants to withstand the drought stress. All of these results are supported by studies on amino acid and metal chelates on Ajwain by Ali *et al*., [36]. Foliar applied various levels of Zn-Asp further increase the concentrations of these compounds. The anthocyanin analysis in the form of free and bound anthocyanin and total anthocyanin contents were also studied. Zn-Asp treatments caused maximum increase in anthocyanin contents. The accumulation of these compounds such as sugars and osmolytes serve as important measure in reducing the hazards of drought constraint and all of these compounds serve as important candidates in mitigating drought stress [42]. The accumulation of soluble sugars in response to water shortage might be due to breakdown of starch. The accumulation of soluble sugars and flavonoids play major part as osmoprotectants therefore these compounds are stress mitigators. There is significant correlation between induction of drought tolerance and accumulation of total soluble sugars [42]. Plants accommodate osmolytes in the form of reducing and non-reducing sugars to support their defense against abiotic stressors as innate behaviour. Current study found that the contents of total soluble sugars, reducing and non-reducing sugars are increased under the influence of drought stress. Above discussion highlights the importance and significance of Zn-Asp and finds it most effective in collation with L-Asp and ZnSO4. Thus, the research outcomes will be very beneficial for increasing yield of maize crop which will assist in coping very fundamental necessity of food and fodder for the indigenous communities of the area.

RETRACTED

## Conclusion

Drought stress is a key yield limiting agent. Current study was aimed to compare the potential of ZnSO_4,_ Zn-Aspartate and L-Aspartate foliar spray as osmoprotectant to combat drought stress in maize plants. Foliar applied 0.5% Zn-Asp increased the activities of SOD and POD enzymes by 28.5% and 33.3% respectively which are antioxidants against osmotic stress. The level of lipids peroxidation product (MDA) declined by 43.9% upon foliar fertigation with 0.5% Zn-Asp. Furthermore the mineral acquisition pattern of maize plants was improved due to foliar applied 0.5% Zn-Asp. Finally the study confers that the use of 0.5% of Zn-Asp treatments as foliar spray prove as better osmolyte in mitigation of drought constraint. However further experimentation in terms of other food crops and other mineral amino acid treatments are recommended. The behaviour of the Zn-Asp in the form of nanoparticles spray may be another subject of interest. The study opens the options for further research in agriculture by interpreting the behaviour of mineral amino acid chelates under water deficit environment.
